# The Correlation between the Level of Skin Advanced Glycation End Products in Type 2 Diabetes Mellitus and the Stages of Diabetic Retinopathy and the Types of Traditional Chinese Medicine Syndrome

**DOI:** 10.1155/2022/5193944

**Published:** 2022-07-08

**Authors:** Senwei Zhang, Ping Ma, Qiu Chen

**Affiliations:** ^1^School of Basic Medicine, Chengdu University of Traditional Chinese Medicine, Chengdu 610072, China; ^2^Department of Microbiology and Immunology, Chengdu University of Traditional Chinese Medicine, Chengdu 610072, China; ^3^Department of Endocrinology, Hospital of Chengdu University of Traditional Chinese Medicine, Chengdu 610072, China

## Abstract

**Objective:**

We aimed to analyze the correlation between the level of skin advanced glycation end products (AGEs) in type 2 diabetes mellitus (T2DM) patients and the diabetic retinopathy (DR) staging in different traditional Chinese medicine (TCM) syndromes.

**Methods:**

416 T2DM patients were divided into normal group, nonproliferative diabetic retinopathy (NPDR) group (mild, moderate, and severe), and proliferative diabetic retinopathy (PDR) group according to the DR grade. Patients' height, weight, fasting blood glucose (FBG), hemoglobin A1C (HbA1c), blood lipid, renal function, and skin AGEs were measured. According to TCM syndrome differentiation criteria, 230 patients with T2DM and DR were divided into I. qi and yin deficiency, collateral stasis group; II. liver and kidney deficiency, eye collaterals loss group; and III. yin and yang deficiency, blood stasis, and phlegm coagulation group.

**Results:**

The skin AGEs levels of different DR staging groups were statistically significant (*P* < 0.05), and the skin AGEs levels in the mild and moderate NPDR groups were significantly higher (*P* < 0.05) than those of the normal group. It was significantly higher (*P* < 0.05) in the severe NPDR group than in the normal group, mild and moderate NPDR groups. The skin AGEs levels of the PDR group were significantly higher (*P* < 0.05) than the normal group, mild and moderate NPDR groups. It was positively correlated with DR stage, HbA1c, total cholesterol (TC), low-density lipoprotein (LDL), and urine metal analysis (UMA) (*r* = 0.467, 0.411, 0.413, 0.503, 0.424, *P* < 0.05). The skin AGEs levels of the qi and yin deficiency and collaterals stasis syndrome group were significantly higher (*P* < 0.05) than in the liver and kidney deficiency and eye collaterals loss groups. It was also significantly higher (*P* < 0.05) in yin and yang deficiency, blood stasis, and phlegm coagulation syndrome groups than in qi and yin deficiency and collaterals stasis syndrome groups.

**Conclusion:**

There is a positive correlation between skin AGEs and DR staging in T2DM patients. Skin AGEs level is predictive for the risk of DR complications in T2DM patients and is vital in assessing DR degree per TCM syndrome type.

## 1. Introduction

Due to the continuous economic progress and improved living conditions, T2DM is spreading rapidly worldwide [1]. In 2009, Yang et al. [2] elaborated detailed data on the epidemiology of more than 40,000 people in 15 provinces in China. Nowadays, the average risk of diabetes for people over 20 years old in China is 9.7%. However, the probability of prediabetes is more than 15.0%.

Diabetes is a metabolic disease caused by hyperglycemia. Its chronic complications spread throughout the body's blood vessels, causing chronic damage to the eyes, kidneys, heart, and nerves. It may cause dysfunction of vital organs and endanger the patient's healthy life. The most common and deadly type of diabetic complications is diabetic microvascular complications caused by microvascular disease. Relevant investigations have shown that the onset of diabetic microvascular complications is due to the damage to microvessels caused by high blood sugar passing through multiple tissues. Hyperglycemia can cause damage to the microvasculature when it passes through multiple tissues, arousing protein kinase C, forming large amounts of glycosylated endpoints, and inducing polyol metabolic pathways and oxidative stress [3–6].

Diabetes microvascular complications are embodied in the skin, nerve, kidney, and other tissues. One of the most common microvascular complications of diabetes is DR, which is a crucial factor in blindness in the world today. Due to the increasing incidence of diabetes, the incidence of diabetic DR is also increasing. Nowadays, more than 90 million people are suffering from DR worldwide. Among them, about 1700 million PDR patients, more than 20 million DME patients, and nearly 30 million DR patients are prone to blindness [7]. It has been proven that diabetes can cause damage to all vital retinal tissues, such as pigmented epithelial tissue, ganglion tissue, Muller tissue, and epithelial tissue. This damage is a relatively cumbersome process, and this system has not been fully explained. The survey on Wisconsin diabetes DR shows that diabetic patients have different degrees of DR after 20 years of illness. Among them, PDR can account for 20.0% of T2DM patients [8]. The onset probability of DR varies from the group with the lowest baseline HbA1c value to the highest group now, and it accounts for about 90.0% in the highest group; it develops from the original simple DR to PDR, which is also related to the baseline HbA1c value. Epidemiological experiments have shown that baseline HbA1c is related to the risk of microvascular complications. When HbA1c is reduced by 1%, microvascular complications will be reduced by 35.0% [9].

AGEs are nonreducible products produced by the free amino groups of nucleic acids, lipids, amino acids, or proteins, and other macromolecular substances and the aldehyde groups of reducing sugars through processes such as oxidation and cleavage without enzyme promotion. AGEs can fuse with various tissues in the human body and damage these tissues, thereby damaging the human body. Experiments show that AGEs can accelerate the aging of the human body and cause various chronic degenerative diseases, such as atherosclerosis, Alzheimer's disease, and diabetes [1, 10, 11]. Therefore, reducing AGEs can slow down the speed of aging and prevent many chronic degenerative diseases. The most crucial change in diabetic DR is the loss of pericytes and the disorder of endothelial cell function, which may cause blockage of capillaries and insufficient blood supply to the retina [12]. There are AGEs in retinal blood vessels and neuroglia. Although they can cause damage to retinal blood vessels, aminoguanidine can prevent this pathological process [13]. It is worth mentioning that aminoguanidine delays the pathological process of diabetic DR, but it cannot stop the initial pathological changes in mice. After AGEs cultivated with calf serum interfered with retinal pericytes, it was found that AGEs immediately became toxic to pericytes, causing its development to slow down, and was related to the concentration of AGEs. AGEs accelerate the death of retinal pericytes through NF-*κ*B activation [14].

Diabetes retinopathy was not known to the public in ancient times. Therefore, most of them were classified into Chinese medicine ophthalmology. According to the guide of traditional Chinese medicine for prevention and treatment of DR, which is issued by China Association of Traditional Chinese Medicine in 2011, TCM syndromes for DR include three types: (1) qi and yin deficiency, collateral stasis (stage I–III DR); (2) liver and kidney deficiency, eye collaterals loss (stage III–IV DR); and (3) yin and yang deficiency, blood stasis, and phlegm coagulation (stage IV–V DR). “Stage DR” is the classification of western medicine. Recent clinical and experimental investigations have shown that TCM effectively prevents and alleviates DR [15–18]. The primary basis of the treatment in TCM is syndrome differentiation. According to syndrome differentiation, TCM has different treatment principles for DR, such as boosting qi and nourishing yin, enriching the liver and kidney, invigorating the spleen and removing dampness, and activating blood and removing stasis, thus unblocking the collaterals. The use of herbs also differs according to these principles [19, 20].

From traditional Chinese medical perspective, diabetes can be induced by weary internal injuries, liver qi stagnation, uncontrolled diet, and exogenous cult poison endowment factors. Pathogenesis mainly includes heated damage, essence loss, blood circulation silt blocking, endogenous phlegm, dark fluid consumption from diabetes, of which “yin deficiency, dryness and heat” is the basic pathogenesis. At present, Chinese medicine has made significant progress in treating diabetes and has much experience in the etiology, pathogenesis, syndrome differentiation, and treatment [21–23].

In the present study, we studied the correlation between skin AGEs and the stages of DR and the types of TCM syndrome.

## 2. Materials and Methods

### 2.1. Participants and Procedures

From 7/2016 to 6/2018, T2DM patients received treatment in the Endocrinology Department. In addition, 416 direct ophthalmoscopy or fundus photography results and skin AGEs in patients with noninvasive test results were recorded.

### 2.2. Inclusion Criteria

(1) Following the 2017 ADA Diabetes Association Standards of Medical Care:
  1. FPG≥126 mg/dL (7.0 mmol/L) (no calorie intake for at least 8 h)
  2. In the OGTT test, the 2- hour blood glucose ≥200 mg/dL (11.1 mmol/L) (75 g anhydrous glucose dissolved in water according to the WHO standard)
  3. Glycated hemoglobin ≥6.5% (48 mmol/mol) (the NGSP certified and standardized DCCT test)
  4. Patients with typical hyperglycemia or hyperglycemic crisis symptoms, random blood glucose ≥200 mg/dL (11.1 mmol/L)
(2) In line with Diabetic Retinopathy Preferred Practice Pattern that is issued by the American Academy of Ophthalmology in 2016: according to the lesions seen under the fundus lens after mydriasis, they are divided into normal: no obvious retinopathy or abnormality; mild NPDR: microaneurysm; moderate NPDR: more serious than microaneurysms, but less severe than NPDR; severe NPDR: any of the following (the 4-2-1 rule) and no signs of proliferative retinopathy.

There were severe intraretinal hemorrhage and microaneurysms in all four quadrants. Identify venous beaded changes in two or more quadrants: moderate IRMA in one or more quadrants. International definition: any of the following with no signs of proliferative retinopathy: more than 20 intraretinal hemorrhages in the four quadrants. Identify venous beaded changes in two or more quadrants: outstanding IRMA in one or more quadrants. PDR : one or both of the following: neovascularization vitreous/subretinal hemorrhage. Any patient with two or more characteristics of severe NPDR is considered to have very severe NPDR.

### 2.3. Exclusion Criteria

1. Diagnosed with type 1 diabetes
2. Those with a history of eye trauma, surgery, and age-related macular degeneration, glaucoma, or retinal diseases other than DR
3. Those who are undergoing hemodialysis treatment and currently suffer from malignant, inflammatory diseases or chronic respiratory diseases
4. The position of the measured skin scarring, lichenification, combined vitiligo, skin abnormalities, and infectious diseases
5. The fundus photography is not checked, or the result of fundus photography is not recorded in the medical history
6. Those who participate in any other clinical research, including any interventional research and any drug clinical research

The T2DM patients who meet the above criteria are divided into normal group, mild NPDR group, moderate NPDR group, severe NPDR group, and PDR group according to the degree of DR.

### 2.4. Determination Assays

1. Measuring height and weight: when measuring height, use cm as the unit, with both arms drooping naturally, heels tight, and the joints naturally opening 60 degree. The heels, shoulders, and sacrum should be close to the uprights, and the body should stand straight. Place the head straight, with the bottom of the eye socket and the top of the tragus in a horizontal position. When measuring the weight: in kg, the person being measured should wear light clothing such as short sleeves and shorts.
2. Measuring FBG: Hitachi 7600 biochemical analyzer is used as the measuring instrument, and the measuring method is the glucose oxidase method. Ningbo Mecang Biotechnology Co., Ltd. supplies kits for the test process.
3. Determination of HbA1c: the instrument is a Norwegian NycoCard Reader II type particular protein quantifier, which uses biochemical chromatography and is equipped with imported initial reagents.
4. Determination of lipid: Hitachi Instruments 7600 biochemical analyzer measured the TC, TG, HDL, or LDL levels.
5. Renal function test: the instrument is Hitachi 7600 biochemical analyzer, which adopts the immune-scattering turbidimetric method to determine urine UMA, and the kit is provided by Beijing Kemei Dongya Biotechnology Co., Ltd.
6. Test skin AGEs : the instrument is a noninvasive detection instrument, AGE Pro, developed by Anhui Yikangda Optoelectronics Technology Co., Ltd., invested and founded by the Biomedical Optics Innovation Team, the Chinese Academy of Sciences. This instrument has a short detection time, no blood draw, and no trauma.

### 2.5. Statistical Analysis

All data analyses have been performed using SPSS 7.0 statistical software, the measurement data of normal or approximately normal distribution is represented by the mean ± standard deviation (x̄ ± *s*), and the data of skewed distribution is represented by the median (interquartile range) [M (Q)]. For comparison between groups, a *t*-test was used for average distribution data, the rank-sum test was used for skew data, and analysis of variance was used for comparison between the three groups. When *P* < 0.05, the LSD-t test was used for further pairwise comparisons, and percentage data were used for count data—using the chi-square test. Correlation analysis was performed using the Pearson-Spearman correlation analysis. *P* < 0.05 is considered statistically significant.

## 3. Results

### 3.1. Comparison of Primary Data of Different DR Staging Groups

There was no significant difference between different DR groups' gender, age, height, and weight (*P* > 0.05). FPG levels were significantly higher (*P* < 0.05) in severe NPDR group than normal and mild NPDR groups. The FPG level in the PDR groups was significantly higher than that of the normal group, which was statistically significant (*P* < 0.05). The HbA1c levels were significantly higher (*P* < 0.05) in the moderate NPDR group than the normal and mild NPDR groups. TC was significantly higher in the severe NPDR group and the PDR group (*P* < 0.05) than normal and mild NPDR groups. LDL levels were significantly higher in the mild NPDR group and the moderate NPDR group (*P* < 0.05) than in the normal group. HDL levels were significantly lower in the mild NPDR group than in the normal group (*P* < 0.05). UMA level in the moderate NPDR group, severe NPDR group, and the PDR group was significantly higher than the normal and mild NPDR group (*P* < 0.05) (Table 1).

### 3.2. Comparison of Skin AGEs Levels in Different DR Staging Groups

The skin AGEs in NPDR group were significantly higher than the normal group (*P* < 0.05). Skin AGEs levels in severe NPDR groups were significantly higher than the normal and mild NPDR groups. The PDR skin AGEs were significantly higher than the normal, mild NPDR group and middle NPDR group. The comparison was statistically significant (*P* < 0.05) (Figure 1, Table 2). The level of skin AGEs is positively correlated with HbA1c, TC, LDL, UMA, and DR staging (Table 3).

### 3.3. Comparison of Basic Data of Different TCM Syndrome Groups

The gender, age, height, weight, course of the disease, FPG, HbA1c, TC, TG, HDL, and UMA of different TCM syndrome groups were not statistically significant (*P* > 0.05). In addition, there was no statistical significance in the liver and kidney deficiency and eye-collateral dystrophy groups. However, the LDL was significantly higher than that of the group with deficiency of both qi and yin and collaterals and stasis syndrome and the group with deficiency of both yin and yang and blood stasis and phlegm coagulation, and the comparison was statistically significant (*P* < 0.05) (Table 4).

### 3.4. Comparison of Skin AGEs Levels in Different TCM Syndrome Groups

The skin AGEs levels in the deficiency of both qi and yin and collaterals and stasis syndrome and the yin and yang deficiency, blood stasis, and phlegm coagulation syndrome groups were significantly higher than those in the liver and kidney deficiency and collateral dysfunction groups, which were statistically significant (*P* < 0.05). In addition, the skin AGEs levels of yin and yang deficiency, blood stasis, and phlegm coagulation syndrome group were significantly higher than those of group with deficiency of both qi and yin and collaterals and stasis, which was statistically significant (*P* < 0.05) (Figure 2, Table 5).

## 4. Discussion

Diabetes emerges in the human body mainly due to the absorption of a large amount of high-fat and carbohydrate foods, which leads to an increase in AGEs in the human body. At the same time, the patient's prolonged hyperglycemia results in an increase in the concentration of glucose and fructose in the human blood, oxidative stress, and the glycolysis reaction also changes, leading to the accumulation of toxicity in the human body. The chemical reaction leads to the cross-linking or reorganization of the protein and fat macromolecules in the carbonyl group, which leads to the increase of AGEs in the human body and damages the related tissues [24]. The emergence of AGEs is mainly due to a nonenzymatic reaction. This chemical reaction is irreversible, so it lacks relevant characteristics to interfere with the target. Therefore, it will be challenging to degrade again during diabetes, even if the blood sugar level of diabetic patients is evident in a short time. However, the AGEs in the human body are still challenging to reach the normal level, and the tissue structure continues to accumulate, which leads to further damage [25], leading to the diabetes metabolic memory [26].

AGEs can affect vascular endothelial cells; induce the production of various protein factors related to inflammation, immunity, and atherosclerosis; and interact with each other to accelerate the pathophysiological changes of blood vessels. At the same time, the permeability of endothelial cells becomes thicker, and the ability of cell proliferation decreases, which will eventually lead to the loss of capillary wall function. Since AGEs may induce capillary cells proliferation, the human visual retinal capillary lumen will continue to shrink, thus blocking the capillary channel, completing a series of gynecologic diseases. DR occurs when the cell basal lamina and matrix were degraded. AGEs can bind receptors to affect VEGF cytokines and then indirectly regulate MMP-9, which can play an essential role in cell migration, angiogenesis, and tissue structure remodeling. *In vivo* experiments showed that hyperglycemia could activate MMP-9 under the action of AGEs and accelerate the apoptosis of retinal capillary cells. According to the experimental data of Charlene E Hafer-Macko et al.[27], the contents of VEGF and AGEs in the vitreous of DR patients will continue to increase. Simultaneously, the increase in VEGF secretion by the cells surrounding the capillaries in diabetic patients' bodies can promote the transmission of TGF-*β* signals, which leads to the appearance of barriers in the retina of patients [28, 29]. In addition, because VEGF can increase the expression ability of VCAM-1, it can promote the formation of blood vessels in the retina. Bansal et al. found that AGEs may be responsible for the induction of oxidative stress through augmenting the PMN-mediated generation of ROS and RNI, which in part induces the development of diabetic pathology [30]. A high glucose environment allows AGEs and their receptor expression levels to rise in the system, resulting in inflammation such glial cells, causing DR lesion diseases [31]. In addition, according to the relevant researchers, experimentally derived AGEs can increase the base of the cells in glial cells, thereby promoting the growth of fibroblasts, enabling DR formation of new blood vessels more quickly, which also contributed to DR important reason for increased [32]. According to the Curtis experiments [33], AGEs can stimulate glial cells in this cell and stimulate fibric acid protein in the cell so that the function of this cell becomes chaotic. According to experiments, the level of AGEs in the skin of diabetic patients in the experiment can reflect the condition of damage to large blood vessels, and there is no substantial relationship between the level of AGEs in serum and damage to large blood vessels [34, 35]. Correlation analysis showed that skin AGEs levels were positively correlated with DR staging and positively correlated with HbA1c, TC, LDL, and UMA. It is suggested that the level of skin AGEs has predictive value for the risk of DR in T2DM patients. The detection of skin AGEs as a convenient, simple, noninvasive, and rapid detection method has significant potential value in the screening and diagnosing of diabetic DR. We also showed a relatively lower expression of AGE in liver and kidney deficiency group than other groups in diabetic patients. A previous study revealed that DR patients of liver and kidney deficiency had lower VEGF and TGF-*β*1 expression after TCM treatment [36]. Vascular endothelial dysfunction may be the pathophysiological basis of liver-kidney yin deficiency syndrome [37]. Combined with the close association of AGE and VEGF as mentioned above in this paragraph, it can be concluded that the relatively lower expression of AGE in liver and kidney deficiency group was associated with the VEGF-mediated vascular endothelial dysfunction.

Chinese medicines are becoming more and more popular due to their health-preserving effects. Clinical and experimental evidence suggest that anti-AGEs-induced damage should be one of the critical reasons [38]. Studies have found that many TCMs such as *Fagopyrum esculentum* Moench [39, 40], Ligusticum Chuanxiong [41], and *Sophora flavescens* [42, 43] exhibit anti-AGEs effects. Tang Youzhi, a master of TCM, believes that the most critical factor of the disease is the simultaneous appearance of qi deficiency and yin deficiency and stagnation. A long time of suffering from the diabetic disease will cause the body to become weak, and the kidneys will gradually lose their essence and energy, which will aggravate the deficiency of qi and blood. Blood coagulation will cause retinal neovascularization over time [44]. Zou Jusheng, a well-known old Chinese doctor in Shanghai, feels that the stomach is hot; the fire burns the body fluid into phlegm, stays, and obstructs the meridians; the veins are stagnant; the evil fire stasis in the body causes body fluid damage; and the blood is not smooth, which causes the blood to flow out of the meridians [45].

There is a direct link between DR TCM symptoms and its clinicopathological features. Zhang Peiran showed that diabetic patients' blood glucose concentration and the average blood glucose levels are not connected. However, TCM directly linked the human body's insufficiency of righteous energy to the visceral dysfunction of blood sugar fluctuations and unstable fluctuations [46]. The most obvious fluctuations in blood sugar are insufficiency of yin fluid and weak yang. Li Zhiying et al. explored the relationship between the symptoms of DR in TCM and visual electrophysiology. The T2DM patients with DR were divided into four types: positive and evil battle each other; insufficient liver and kidney Yin Ye; yang weak, weak spleen; and blood coagulation. The authors found that positive and evil battle each other and blood coagulation was the basic symptom; Dr. Zhangya Xin revealed that there is a direct correlation between the course of diabetes and the type of DR [47]. The traditional concept of Chinese ophthalmology, the “five-wheel theory,” believes that the pupil belongs to the water wheel and directly connects with the kidney. In addition, it also shows that HbA1c is related to the level of DR phlegm-dampness syndrome and dry heat syndrome in the body, and the UMA level is related to the level of Yang Qi weak phlegm-dampness syndrome in DR patients. In the pathological mechanism of diabetes, the poisonous evil is deeply buried and cannot leak out an essential part of it. Toxins are caused by the dysfunction of the viscera, qi, and blood, which causes the meridians to be blocked, and the metabolism of water and fluid is abnormal, leading to the production of stasis and dampness phlegm and other pathogens. It is both a pathological product and a new pathogenic factor.

According to TCM, AGEs can also be classified as “toxins.” Then the relationship between AGEs and the pathogenesis of DR in TCM is worthy of discussion, and understanding the relationship has far-reaching significance for the pathogenesis of diabetic DR and TCM diagnosis and treatment. At present, there are few research reports on the relationship between AGEs and TCM syndrome types, and there are still controversies. Some scholars believe that AGEs have a damaging effect on vascular endothelial cells, and the pathogenesis of deficiency of both qi and yin in traditional Chinese medicine is also reflected in the damage of vascular endothelial cells. Therefore, we speculated that AGEs are related to the pathogenesis of “a deficiency of both qi and yin and stasis of collaterals.”

## 5. Conclusion

This study showed that yin deficiency, skin collaterals, and stagnation group AGEs are significantly higher in liver and kidney deficiency. The AGEs levels were significantly higher in the dystrophy syndrome group, the yin and yang, and blood stasis syndrome group than in the group with deficiency of both qi and yin and collaterals and stasis. It can be seen that patients with yin and yang deficiency, blood stasis, and phlegm coagulation syndrome usually have more severe DR, and the corresponding skin AGEs level is also higher. In conclusion, according to TCM type, skin AGEs levels could significantly determine the DR degree.

## Figures and Tables

**Figure 1:** Skin AGEs levels in different DR stages.

**Figure 2:** Skin AGEs levels in different TCM syndrome groups.

**Table 1:** Comparison of primary data of different DR staging groups.

	Normal group (*n* = 186)	Mild NPDR group (*n* = 114)	Middle NPDR group (*n* = 68)	Severe NPDR group (*n* = 27)	PDR group (*n* = 21)
Gender (male/female)	119/67	63/51	39/29	17/10	14/7
Age (years) [M (Q)]	56.8 (7.4)	59.8 (7.7)	57.5 (9.4)	65.5 (5.1)	62.8 (6.0)
Height (cm)	163.3 ± 5.7	161.8 ± 6.9	163.0 ± 7.5	162.3 ± 7.1	155.3 ± 6.8
Weight (kg)	66.1 ± 4.8	68.9 ± 5.0	66.4 ± 6.4	64.0 ± 6.4	58.0 ± 7.5
Course of disease (year)	3.0 ± 1.6	3.5 ± 1.8	3.4 ± 1.1	3.5 ± 1.5	3.3 ± 1.7
FPG (mmol/L)	9.4 ± 1.4	9.7 ± 1.9	10.2 ± 1.6	11.7 ± 2.8	10.5 ± 2.1
HbA1c (%)	8.7 ± 1.7	8.5 ± 1.6	9.2 ± 2.0	8.7 ± 2.1	9.2 ± 1.7
TC (mmol/L)	4.4 ± 1.7	4.7 ± 1.6	4.5 ± 1.3	5.5 ± 1.4	5.1 ± 2.7
TG (mmol/L)	1.3 ± 0.7	1.5 ± 0.7	1.7 ± 0.8	2.0 ± 0.4	1.3 ± 0.5
LDL (mmol/L)	2.1 ± 0.8	2.7 ± 0.9	2.7 ± 0.5	2.5 ± 0.8	2.2 ± 1.1
HDL (mmol/L)	1.5 ± 0.8	1.1 ± 0.5	1.4 ± 0.9	1.3 ± 0.5	1.4 ± 0.4
UMA (g/L)	42.6 ± 7.5	70.8 ± 9.5	126.6 ± 23.2	315.7 ± 37.5	298.6 ± 64.8

**Table 2:** Comparison of skin AGEs levels in different DR staging groups.

Group	AGEs
Normal group (*n* = 186)	90.1 ± 13.8
Mild NPDR group (*n* = 114)	93.0 ± 17.3
Middle NPDR group (*n* = 68)	93.5 ± 15.5
Severe NPDR group (*n* = 27)	104.8 ± 14.8
PDR group (*n* = 21)	104.0 ± 9.5
*F*	21.046
*P*	<0.001

**Table 3:** Correlation analysis between skin AGEs levels and various indicators.

Index	Correlation analysis	Correlation coefficient	*P*
HbA1c	Pearson	0.511	<0.01
TC	Pearson	0.463	<0.01
LDL	Pearson	0.502	<0.01
UMA	Pearson	0.411	<0.01
DR staging	Spearman	0.467	<0.01

**Table 4:** Comparison of basic data of different TCM syndrome groups.

	Qi and yin deficiency, collateral and vessel stasis syndrome group (*n* = 72)	Liver and kidney deficiency, eye and collateral dystrophy syndrome group (*n* = 99)	Yin and yang deficiency, blood stasis and phlegm coagulation group (*n* = 59)
Gender (male/female)	39/33	60/39	34/25
Age (year) [M (Q)]	59.5 (8.1)	57.4 (9.2)	59.5 (8.8)
Height (cm)	162.9 ± 4.9	160.6 ± 8.3	162.6 ± 6.8
Wight (kg)	64.7 ± 6.0	67.6 ± 7.3	66.9 ± 7.5
The course of disease (year)	3.3 ± 1.7	3.4 ± 1.5	3.6 ± 1.6
FPG (mmol/L)	9.6 ± 1.8	9.6 ± 1.3	9.5 ± 1.7
HbA1c (%)	8.6 ± 1.9	9.0 ± 1.4	8.9 ± 1.5
TC (mmol/L)	4.6 ± 1.5	4.5 ± 1.8	4.5 ± 1.8
TG (mmol/L)	1.6 ± 0.5	1.6 ± 0.7	1.5 ± 0.6
LDL (mmol/L)	2.4 ± 0.8	2.8 ± 0.6	2.5 ± 0.9
HDL (mmol/L)	1.3 ± 0.9	1.2 ± 0.4	1.1 ± 0.5
UMA (g/L)	85.9 ± 13.2	79.4 ± 18.4	95.36 ± 33.8

**Table 5:** Comparison of skin AGEs levels in different TCM syndrome groups.

Group	AGEs
Deficiency of qi and yin deficiency, collateral and vessel stasis syndrome (*n* = 72)	93.5 ± 3.6
Deficiency of liver and kidney deficiency, dystrophy of eye and collaterals (*n* = 99)	90.1 ± 4.2
Yin and yang deficiency, blood stasis and phlegm coagulation syndrome (*n* = 59)	97.7 ± 3.1
*F*	23.267
*P*	<0.001

## Data Availability

All data included in the present study are listed in the article.

## References

[1] Lai M. C., Liu W. Y., Liou S. S., Liu I. M. (2022). The citrus flavonoid hesperetin encounters diabetes-mediated alzheimer-type neuropathologic changes through relieving advanced glycation end-products inducing endoplasmic reticulum stress. *Nutrients*.

[2] Yang W., Lu J., Weng J. (2010). Prevalence of diabetes among men and women in China. *New England Journal of Medicine*.

[3] Stumvoll M., Goldstein B. J., van Haeften T. W. (2005). Type 2 diabetes: principles of pathogenesis and therapy. *Lancet*.

[4] Kitabchi A. E., Umpierrez G. E., Miles J. M., Fisher J. N. (2009). Hyperglycemic crises in adult patients with diabetes. *Diabetes Care*.

[5] Giacco F., Brownlee M. (2010). Oxidative stress and diabetic complications. *Circulation Research*.

[6] Faselis C., Katsimardou A., Imprialos K., Deligkaris P., Kallistratos M., Dimitriadis K. (2020). Microvascular complications of type 2 diabetes mellitus. *Current Vascular Pharmacology*.

[7] Yau J. W., Rogers S. L., Kawasaki R. (2012). Global prevalence and major risk factors of diabetic retinopathy. *Diabetes Care*.

[8] Arevalo J. F., Lasave A. F., Wu L. (2017). Intravitreal bevacizumab for proliferative diabetic retinopathy: results from the pan-American collaborative retina study group (pacores) at 24 months of follow-up. *Retina*.

[9] Stratton I. M., Adler A. I., Neil H. A. (2000). Association of glycaemia with macrovascular and microvascular complications of type 2 diabetes (UKPDS 35): prospective observational study. *BMJ*.

[10] Wang Z. Q., Jing L. L., Yan J. C. (2018). Role of AGEs in the progression and regression of atherosclerotic plaques. *Glycoconjugate Journal*.

[11] Singh R., Barden A., Mori T., Beilin L. (2001). Advanced glycation end-products: a review. *Diabetologia*.

[13] Wannamethee S. G., Welsh P., Papacosta O. (2017). Circulating soluble receptor for advanced glycation end product: cross-sectional associations with cardiac markers and subclinical vascular disease in older men with and without diabetes. *Atherosclerosis*.

[14] Kim J., Jo K., Lee I. S., Kim C. S., Kim J. S. (2016). The extract of aster koraiensis prevents retinal pericyte apoptosis in diabetic rats and its active compound, chlorogenic acid inhibits AGE formation and AGE/RAGE interaction. *Nutrients*.

[15] Behl T., Kotwani A. (2017). Chinese herbal drugs for the treatment of diabetic retinopathy. *Journal of Pharmacy and Pharmacology*.

[16] He L., Wang H., Gu C., He X., Zhao L., Tong X. (2016). Administration of traditional Chinese blood circulation activating drugs for microvascular complications in patients with type 2 diabetes mellitus. *Journal of Diabetes Research*.

[17] Pang B., Zhou Q., Zhao T. Y. (2015). Innovative thoughts on treating diabetes from the perspective of traditional Chinese medicine. *Evidence Based Complementary Alternative Medicine*.

[18] Zhang H. W., Zhang H., Grant S. J., Wan X., Li G. (2018). Single herbal medicine for diabetic retinopathy. *Cochrane Database of Systematic Reviews*.

[19] PingPing X., Xu W. (2014). Research progress on traditional Chinese medicine treatment of diabetic retinopathy. *China Journal of Traditional Chinese Medicine and Pharmacy*.

[20] Zhao Y.-Q., Li Q.-S., Xiang M.-H., Zhang W., Zhang X.-R. (2017). Distribution of traditional Chinese medicine syndromes of diabetic retinopathy and correlation between symptoms. *China journal of Chinese materia medica*.

[21] Wang J., Ma Q., Li Y. (2020). Research progress on traditional Chinese medicine syndromes of diabetes mellitus. *Biomedicine & Pharmacotherapy*.

[22] Dou Z., Xia Y., Zhang J. (2021). Syndrome differentiation and treatment regularity in traditional Chinese medicine for type 2 diabetes: a text mining analysis. *Frontiers in Endocrinology*.

[23] Yan X. F., Ni Q., Wei J. P., Lin L. (2014). A systematic review and meta-analysis of type 2 diabetes mellitus treatment based on the “three-typed syndrome differentiation” theory in Chinese medicine. *Chinese Journal of Integrative Medicine*.

[24] Nowotny K., Jung T., Höhn A., Weber D., Grune T. (2015). Advanced glycation end products and oxidative stress in type 2 diabetes mellitus. *Biomolecules*.

[25] Mastrocola R., Nigro D., Chiazza F. (2016). Fructose-derived advanced glycation end-products drive lipogenesis and skeletal muscle reprogramming via SREBP-1c dysregulation in mice. *Free Radical Biology and Medicine*.

[26] Ceriello A. (2012). The emerging challenge in diabetes: the “metabolic memory”. *Vascular Pharmacology*.

[27] Hafer-Macko C. E., Ivey F. M., Gyure K. A., Sorkin J. D., Macko R. F. (2002). Thrombomodulin deficiency in human diabetic nerve microvasculature. *Diabetes*.

[28] Kim J., Kim C. S., Sohn E., Jeong I. H., Kim H., Kim J. S. (2011). Involvement of advanced glycation end products, oxidative stress and nuclear factor-kappaB in the development of diabetic keratopathy. *Graefes Archive for Clinical and Experimental Ophthalmology*.

[29] Rodriguez R., Lowe K., Keniry M., Tsin A. (2021). Involvement of TGF*β* signaling pathway in oxidative stress and diabetic retinopathy. *Archives of Clinical and Experimental Ophthalmology*.

[30] Bansal S., Siddarth M., Chawla D., Banerjee B. D., Madhu S. V., Tripathi A. K. (2012). Advanced glycation end products enhance reactive oxygen and nitrogen species generation in neutrophils in vitro. *Molecular and Cellular Biochemistry*.

[31] Zong H., Ward M., Madden A. (2010). Hyperglycaemia-induced pro-inflammatory responses by retinal Müller glia are regulated by the receptor for advanced glycation end-products (RAGE). *Diabetologia*.

[32] Wang S. (2007). Overview of the research on the treatment of diabetes in traditional Chinese medicine. *Henan traditional chinese medicine*.

[33] Zhao H. (2009). Longevity and life preservation treating destructive thirst experience. *Guang ming zhong yi*.

[34] Liu X., Chen L., Dong L. (2007). Pathogenesis of type 2 diabetes. *World journal of integrated traditional and western medicince*.

[35] Han Y., Zhang L., Qiu X. (2010). Discussion on the etiology and pathogenesis of diabetes from “heat poison”. *Guang ming zhong yi*.

[36] Liu R., Yuan F., Gong C. (2021). Clinical efficacy of jiawei qiju dihuang decoction in the treatment of patients with diabe etic nephropathy with yin deficiency syndrome of liver and kidney combined with blood stasis and influence on serum VEGFIGF-1 and TGF-31 levels. *World Journal of Integrated Traditional and Western Medicine*.

[37] Zhou Y., Lan X. (2010). Relationship between liver-kidney rin deficiency and vascular endothelial dysfunction. *Acta Chinese Medicine and Pharmacology*.

[38] Zhang W., Zhao T., Zhao Y., Gui D., Xu Y. (2020). Advanced glycation end products in Chinese medicine mediated aging diseases: a review. *Current Vascular Pharmacology*.

[39] Zhang C., Teng F., Tu J., Zhang D. (2014). Ultrasound-enhanced protective effect of tetramethylpyrazine against cerebral ischemia/reperfusion injury. *PLoS One*.

[40] Lei Y., Yang J., Zhao H. (2010). Experimental study on extracts from ginseng, notoginseng and chuanxiong for delaying vascular aging in senescent mice. *Zhongguo Zhong Xi Yi Jie He Za Zhi*.

[41] Zheng Q., Huang Y. Y., Zhu P. C. (2018). Ligustrazine exerts cardioprotection in animal models of myocardial ischemia/reperfusion injury: preclinical evidence and possible mechanisms. *Frontiers in Pharmacology*.

[42] Pashikanti S., de Alba D. R., Boissonneault G. A., Cervantes-Laurean D. (2010). Rutin metabolites: novel inhibitors of nonoxidative advanced glycation end products. *Free Radical Biology and Medicine*.

[43] Khajevand-Khazaei M. R., Mohseni-Moghaddam P., Hosseini M., Gholami L., Baluchnejadmojarad T., Roghani M. (2018). Rutin, a quercetin glycoside, alleviates acute endotoxemic kidney injury in C57BL/6 mice via suppression of inflammation and up-regulation of antioxidants and SIRT1. *European Journal of Pharmacology*.

[44] Lin L., Wang E., Yuan H., Chen L. (2009). Treating diabetes by soothing liver and strengthening spleen. *Guang ming zhong yi*.

[45] Arsov S., Graaff R., van Oeveren W. (2014). Advanced glycation end-products and skin autofluorescence in end-stage renal disease: a review. *Clinical Chemistry and Laboratory Medicine*.

[46] Hartog J. W., Hummel Y. M., Voors A. A. (2008). Skin-autofluorescence, a measure of tissue advanced glycation end-products (AGEs), is related to diastolic function in dialysis patients. *Journal of Cardiac Failure*.

[47] Meerwaldt R., Hartog J. W., Graaff R. (2005). Skin autofluorescence, a measure of cumulative metabolic stress and advanced glycation end products, predicts mortality in hemodialysis patients. *Journal of the American Society of Nephrology*.

